# Research on UCAV Maneuvering Decision Method Based on Heuristic Reinforcement Learning

**DOI:** 10.1155/2022/1477078

**Published:** 2022-03-03

**Authors:** Wang Yuan, Zhang Xiwen, Zhou Rong, Tang Shangqin, Zhou Huan, Ding Wei

**Affiliations:** ^1^Air Force Engineering University, Xi'an, China; ^2^Southeast University, Nanjing, China

## Abstract

With the rapid development of unmanned combat aerial vehicle (UCAV)-related technologies, UCAVs are playing an increasingly important role in military operations. It has become an inevitable trend in the development of future air combat battlefields that UCAVs complete air combat tasks independently to acquire air superiority. In this paper, the UCAV maneuver decision problem in continuous action space is studied based on the deep reinforcement learning strategy optimization method. The UCAV platform model of continuous action space was established. Focusing on the problem of insufficient exploration ability of Ornstein–Uhlenbeck (OU) exploration strategy in the deep deterministic policy gradient (DDPG) algorithm, a heuristic DDPG algorithm was proposed by introducing heuristic exploration strategy, and then a UCAV air combat maneuver decision method based on a heuristic DDPG algorithm is proposed. The superior performance of the algorithm is verified by comparison with different algorithms in the test environment, and the effectiveness of the decision method is verified by simulation of air combat tasks with different difficulty and attack modes.

## 1. Introduction

From a macro point of view, air combat decision making refers to one party in air combat providing corresponding control instructions to fighter jets after analyzing and judging battlefield information so that it can complete the dominant attack position occupying the enemy. Decision making is the core of air combat, and its rationality will determine the final outcome of air combat [1].

In recent years, with the continuous improvement and development of deep learning (DL) theory, the deep reinforcement learning (DRL) algorithm combined with deep learning and reinforcement learning has become a research hotspot in artificial intelligence. With no training samples, not limited by specific models, and able to take into account the long-term impact of actions and other advantages, deep reinforcement learning methods have gradually received attention in the research of air combat maneuver decision making. Deep reinforcement learning can be divided into two types: value-based reinforcement learning algorithms and policy-based reinforcement learning algorithm. [2–4].

Watkins proposed Q learning on the basis of dynamic programming, which forms the evaluation value of each state action through repeated experiments and iterations. However, due to the limitation of the look-up table method, its algorithm is only applicable to the applications of finite state space and action space. Subsequently, with the increasing dimension of the state space of the research object, DNNs, CNNs, or RNNs were used to replace the action value function *Q*, forming the deep *Q* network algorithm (DQN) [5, 6] and introducing the experience replay target q-value network. In reference [7], the DQN algorithm is used to construct autonomous obstacle avoidance decisions for UAVs. By transforming the obstacle avoidance process of UAVs into a Markov decision problem and introducing neural networks for the decision model and improving the replay process, random dynamic obstacle avoidance of UCAVs in a 3D environment is realized, which effectively improves the efficiency of task execution. The DeepMind team realized autonomous learning in the Openai Gym simulation platform based on the DQN algorithm [8] and won the battle with professional players with absolute results, which again proved that DQN has obvious advantages over traditional algorithms and humans in decision-making ability. Subsequently, the AlphaGO System and the AlphaGO Master were developed and used to defeat all the world champions, which caused a sensation and made people reunderstand artificial intelligence technology. In 2017, AlphaGo Zero realized a self-game, started training without task samples, and further improved both speed and effect. Silver et al. [9] and Liu and Ma [10] constructed a discrete UAV maneuvering action library and realized the autonomous attack of a low-dynamic UAV by using a DQN. In reference [11], the DQN algorithm is used in UAV air combat confrontation, and the min-max algorithm is used to solve value functions in different states. The simulation result verifies that this method has good effects.

Value-based reinforcement learning methods cannot deal with the problem of continuous action space [12–15]. Lillicrap combined the deterministic policy gradient algorithm [16] and actor-critic framework, and a deep deterministic policy gradient (DDPG) algorithm is proposed to address continuous state space and continuous action space problems [17].

Wang et al. used the DDPG algorithm to study the pursuit strategy of a car in a plane. [18] Yang used the DDPG algorithm to construct an air combat decision system. Focusing on the problem of low data utilization due to the lack of prior knowledge of air combat in the DDPG algorithm, they proposed adding the sample data of the existing mature maneuvering decision-making system into the replay buffer in the initial training stage to prevent the DDPG algorithm from falling into a local optimum during training. Thus, the convergence speed of the algorithm was accelerated. [19].

At present, deep reinforcement learning has been widely applied in unmanned vehicle control, [20] robot path planning and control, [21] pursuit and avoidance of targets, [22] unmanned driving [23, 24], and real-time strategy games [25, 26]. However, most of the reinforcement learning algorithms used in air combat maneuvering decision making are discrete action space algorithms, which inevitably face the problems of rough flight paths and limited reachable domains. At the same time, model-free deep reinforcement learning algorithms are widely used at present, which are capable of self-learning effective air combat maneuver strategies independent of human air combat expert experience and have a general learning framework. However, model-free deep reinforcement learning algorithms need to interact with the environment to obtain a large number of training samples, and inefficient data utilization and learning efficiency become important bottlenecks in the practical application of model-free reinforcement learning methods. [3, 27–30].

According to the above problems, in this paper, the UCAV maneuvering decision-making problem in continuous action space is studied. By introducing a heuristic exploration strategy, the problem of insufficient exploration strategy exploration ability and low data utilization in the DDPG algorithm is improved, and then a UCAV air combat maneuver decision-making method based on the heuristic DDPG algorithm is proposed.

## 2. Air Combat Environment Design

### 2.1. Flight Motion Model

To consider the coupling relationship between the control quantities when continuous control quantities are independently sought, the UCAV platform model based on the angle of attack, engine thrust, and roll angle as control quantities is adopted to fully consider the influence of the aerodynamic characteristics of the platform on the flight state so that the model is closer to reality and the flight trajectory is more realistic, increasing its engineering use value. Its three-degree-of-freedom mass kinematic model is as follows:

(1) $$\begin{array}{c} \left\{\begin{array}{c} \dot{x}=v\;\cos\;\gamma \;\cos\;\psi ,\\ \dot{y}=v\;\cos\;\gamma \;\sin\;\psi ,\\ \dot{z}=v\;\sin\;\gamma , \end{array}\right) \end{array}$$

where $\dot{x}$, $\dot{y}$, and $\dot{z}$ are the components of the velocity of the UCAV in the inertial coordinate system. *γ* represents the flight path angle, and *ψ* represents the yaw angle.

The updated equations for its velocity *v*, flight path angle *γ*, and yaw angle *ψ*, i.e., the particle dynamics model, are as follows:

(2) $$\begin{array}{c} \left\{\begin{array}{c} \dot{v}=\frac{T\;\cos\;\alpha -D}{m}-g\;\sin\;\gamma ,\\ \dot{\gamma }=\frac{\left(L+T\;\sin\;\alpha \right)\cos\;\phi }{mv}-\frac{g}{v}\cos\;\gamma ,\\ \dot{\psi }=\frac{\left(L+T\;\sin\;\alpha \right)\sin\;\phi }{mv\;\cos\;\gamma }, \end{array}\right) \end{array}$$

where *m* is the mass of the UCAV, *g* is the acceleration of gravity, *D* is the drag parameter, and *T*, *α*, and *ϕ* are the three control quantities of the model, that is, the angle of attack, engine thrust, and roll angle, respectively.

As seen from the above equation, to obtain a direct mapping relationship between the model control quantities *u*=[*T*, *α*, *ϕ*] and the state change, the drag parameter *D*, the lift parameter *L*, and the thrust *T* need to be solved; however, as the drag, lift, and thrust are influenced by various factors, such as altitude, atmospheric density, aerodynamic shape, and flight speed, and are strongly coupled and nonlinear, their parameter expressions are difficult to derive through traditional mechanics. In this paper, the relevant aerodynamic parameters of a publicly available storm shadow UAV [31] are fitted by a BP neural network [32–35] to determine the important aerodynamic and dynamic characteristics, with the aim of establishing a more detailed and realistic model of the UCAV platform, which will provide the basis for subsequent maneuvering decision making in continuous action space.

### 2.2. Geometry of Air Combat

When describing the geometric relationship between aircraft in air combat, the important factors usually considered are the distance between two aircraft, heading crossing angle (HCA), line of sight (LOS), antenna train angle (ATA), and aspect angle (AA). The distance between two aircraft is usually expressed by the calculation *R*=norm(*x*_*e*_ − *x*, *y*_*e*_ − *y*, *z*_*e*_ − *z*), which is an important factor to evaluate the air combat situation and judge the launching conditions of weapons. HCA refers to the angle formed by two aircraft courses. LOS is the line between the UCAV and the enemy aircraft. AA refers to the included angle between the LOS and the direction of the enemy aircraft, which represents the angle relation between our aircraft and the enemy under the current attitude. When AA = 180, it indicates that our aircraft is on the extension line of the axis direction of the enemy aircraft's body; that is, the nose of the enemy aircraft is facing our aircraft. ATA refers to the included angle between the sighting line vector and the pointing direction of the axis of the aircraft body and represents the angle relation between the enemy aircraft and the current attitude of the aircraft. ATA = 0° when the enemy aircraft is directly in front of the nose of the aircraft. The above geometric relationship between the enemy and us is shown in Figure 1.

ATA and AA can be expressed as

(3) $$\begin{array}{c} \text{ATA}=\arccos\frac{R\times V_{u}}{\left\|R\right\|\times \left\|V_{u}\right\|},\text{ATA}\in \left[0,\pi \right],\\ \text{AA}=\pi -\arccos\frac{R\times V_{e}}{\left\|R\right\|\times \left\|V_{e}\right\|},\text{AA}\in \left[0,\pi \right]. \end{array}$$

### 2.3. Reward Shaping

The objective of maneuver decisions in close air combat based on reinforcement learning is to find an optimal maneuver strategy to enable the UCAV to complete the attack position to maximize the current cumulative reward. Reward is the only quantitative index of strategy evaluation, which determines the final learning strategy of an agent and directly affects the convergence and learning speed of the algorithm. When the UCAV conducts air combat decision making through deep reinforcement learning, except for the reward for completing the task, there is no reward in the middle process, and there is the problem of sparse reward. Therefore, it is not only necessary to design the reward for completing the task but also crucial to design the guiding reward for each step in each round. In this paper, a reward function including angle, height, distance, and speed factors is designed.

#### 2.3.1. Angle Factor

When the maximum firing range of the UCAV weapon is superior to that of the enemy, the UCAV missile firing conditions can be preferentially met in the head-on encounter with the enemy. Due to the omnidirectional attack capability of the fourth-generation short-range air-to-air missile, there is no need to consider the attitude of the enemy at this time. Therefore, under the current weapon advantage, the angle factor is mainly determined by the ATA of the UCAV. As long as the ATA angle is within the range of the maximum off-axis launch angle, the angle reward can be obtained, specifically expressed as

(4) $$\begin{array}{c} \text{if}\;L_{\max}^{u}>L_{\max}^{e}:\\ r_{A-\text{FRO}}^{t}\left(s_{t}\right)=\left\{\begin{array}{cc} 1, & \text{ATA}\leq \theta_{\max}^{u},\\ -1, & \text{others,} \end{array}\right) \end{array}$$

where *L*_max_^*u*^ is the maximum launching distance of the UCAV airborne weapon, *L*_max_^*e*^ is the maximum launching distance of the enemy aircraft weapon, and *θ*_max_^*u*^ is the maximum off-axis launching angle of the UCAV airborne missile.

When the maximum firing distance of the UCAV weapon is weaker than that of enemy aircraft, it is extremely detrimental to UCAV security. At this time, to ensure their own safety, UCAV should be guided to give full play to their maneuverability and always be located beyond the maximum off-axis angle of enemy aircraft and attack enemy aircraft as far as possible with the tactics of tail attack. In this case, the angle factor should consider both the ATA of the UCAV and AA of the enemy aircraft, and the angle factor design is as follows:

(5) $$\begin{array}{c} if\;L_{\max}^{u}<L_{\max}^{e}:r_{A-\text{BAC}}^{t}\left(s_{t}\right)=\left\{\begin{array}{cc} 1, & \begin{array}{c} \text{if ATA}\leq \theta_{\max}^{u},\\ \frac{\pi }{2}\leq AA, \end{array}\\ 0, & \text{if AA}\leq \frac{\pi }{2},\\ -1, & \text{if others,} \end{array}\right) \end{array}$$

where *L*_max_^*u*^ is the maximum launching distance of the UCAV airborne weapon, *L*_max_^*e*^ is the maximum launching distance of the enemy aircraft weapon, and *θ*_max_^*u*^ is the maximum off-axis launching angle of the UCAV airborne missile.

#### 2.3.2. Height Factor

The height factor not only represents the relationship between the two in the vertical plane in the geometry situation of air combat but also measures the energy advantage of the UCAV. The side that satisfies the height advantage not only has the advantage of energy mobility but can also exert the missile's larger attack range. A high reward factor is achieved when the UCAV is in the desired altitude range relative to the enemy aircraft:

(6) $$\begin{array}{c} r_{H}^{t}\left(s_{t}\right)=\left\{\begin{array}{cc} 1, & \Delta H_{\text{down}}\leq \Delta H\leq \Delta H_{\text{up}},\\ -1, & \text{others,} \end{array}\right) \end{array}$$

where Δ*H*=*z*_*u*_ − *z*_*e*_ represents the relative height of the UCAV and the enemy aircraft, Δ*H*_up_ is the upper limit of maintaining the altitude advantage, and Δ*H*_down_ is the lower limit of maintaining the altitude advantage.

#### 2.3.3. Distance Factor

Distance is an important factor for UCAV platform situation assessment and weapon launch conditions. When the relative distance between two aircraft meets the maximum missile launch distance, the maximum distance factor can be obtained, which is defined as

(7) $$\begin{array}{c} r_{R}^{t}\left(s_{t}\right)=\left\{\begin{array}{cc} 1, & L_{\min}^{u}\leq R_{\text{LOS}}\leq L_{\max}^{u},\\ -1, & \text{others,} \end{array}\right) \end{array}$$

where *R*_LOS_=norm[*x*_*e*_ − *x*_*u*_, *y*_*e*_ − *y*_*u*_, *z*_*e*_ − *z*_*u*_] and *L*_max_^*u*^ and *L*_min_^*u*^ are the maximum and minimum firing ranges of UCAV airborne weapons, respectively.

#### 2.3.4. Speed Factor

When the distance between the two planes reaches the maximum launching distance of the missile, the UCAV sees the speed of the enemy aircraft as the best attack speed. When the distance between the two planes is relatively far, the UCAV should maintain a large flight speed to rapidly form a favorable situation and maintain a kinetic energy advantage with the help of high speed and maneuverability. The speed factor is established as follows:

(8) $$\begin{array}{c} r_{V}^{t}\left(s_{t}\right)=\left\{\begin{array}{cc} 1, & L_{\min}^{u}\leq R_{\text{LOS}}\leq L_{\max}^{u}\cap |\Delta v|\leq \delta_{v},\\ 0.5, & R_{\text{LOS}}\leq L_{\min}^{u}\cap v_{u}>v_{e},\\ 0.5, & R_{\text{LOS}}\geq L_{\max}^{u}\cap v_{u}>v_{e},\\ -1, & \text{others,} \end{array}\right) \end{array}$$

where Δ*v*=*v*_*u*_ − *v*_*e*_ represents the relative speed of the UCAV and enemy aircraft and *δ*_*v*_ is the allowable relative speed difference from the optimal attack speed.

#### 2.3.5. Environmental Factor

When the UCAV air combat strategy is learned through reinforcement learning, in addition to making the UCAV capable of attacking enemy aircraft, the more important prerequisite is that the UCAV has the ability to adapt to the battlefield environment and maintain a safe flight altitude. Therefore, to train the air combat strategy with both air combat capability and safe flight capability, it is necessary to set negative returns in the form of punishment for dangerous flight maneuvers, so the environmental factor *r*_ENV_^*t*^ is constructed as follows:

(9) $$\begin{array}{c} r_{\text{ENV}}^{t}=\left\{\begin{array}{cc} -50, & \left(x_{u},y_{u},z_{u},v_{u}\right)\notin \left(x_{\text{limit}},y_{\text{limit}},z_{\text{limit}},v_{\text{limit}}\right),\\ 0, & \text{others,} \end{array}\right) \end{array}$$

where *x*_limit_=[*x*_min_, *x*_max_],*y*_limit_=[*y*_min_, *y*_max_], and *z*_limit_=[*h*_min_, *h*_max_] represent the range of the operational airspace on the *X*, *Y*, and *Z* axes of the inertial coordinate system, and *v*_limit_=[*v*_min_, *v*_max_] represents the extreme value of the safe flight speed of the UCAV.

#### 2.3.6. End Factor

(10) $$\begin{array}{c} r_{\text{END}}^{t}=\left\{\begin{array}{cc} 100, & \text{if End}=\text{Win,}\\ -100, & \text{if End}=\text{Loss,}\\ 0, & \text{others,} \end{array}\right) \end{array}$$

where End is the result of outcome determination. When the angle, height, distance, and speed reward factors of the UCAV are 1 at the same time, the weapon launch condition is reached, and the UCAV is judged to win, where End can be expressed as

(11) $$\begin{array}{c} \text{End}\left(t\right)=\left\{\begin{array}{cc} \text{Win,} & \text{if }r_{A}^{t}=\left\{\begin{array}{cc} r_{A-\text{FRO}}^{t}\left(s_{t}\right), & \text{if }L_{\max}^{u}>L_{\max}^{e}\\ r_{A-\text{BAC}}^{t}\left(s_{t}\right), & \text{if }L_{\max}^{u}<L_{\max}^{e} \end{array}\right\}=r_{R}^{t}=r_{H}^{t}=r_{V}^{t}=1,\\ \text{Loss,} & \text{if enemy win.} \end{array}\right) \end{array}$$

#### 2.3.7. Total Reward Function

Based on the above analysis, the total reward function is

(12) $$\begin{array}{c} r_{t}\left(s_{t}\right)=\left\{\begin{array}{cc} r_{A-\text{FRO}}^{t}\left(s_{t}\right), & \text{if}L_{\max}^{u}>L_{\max}^{e}\\ r_{A-\text{BAC}}^{t}\left(s_{t}\right), & \text{if}L_{\max}^{u}<L_{\max}^{e} \end{array}\right\}+r_{H}^{t}+r_{R}^{t}+r_{V}^{t}+r_{\text{ENV}}^{t}+r_{\text{END}}^{t}. \end{array}$$

## 3. Heuristic DDPG Algorithm

This section constructs an exploration strategy that is more effective than traditional Gaussian noise or OU noise. At present, the traditional exploration strategy such as OU usually acts directly on the actions of the strategy network output and makes the actions randomly disturbed in the form of addition to realize the exploration of unknown space. In an air combat environment, unmanned combat aircraft control the amount of high dimensionality and large amplitude range; therefore, the DDPG algorithm is based on the strategy of OU explores noise and is likely to create many blind spots in the search. The serious influence training effect, at the same time, is based on the limited performance and flight safety, UCAV variation and volume control of each dimension has a strict limit. When the output action of the policy network is close to the boundary of its scope, it is blind and ineffective to implement exploration by adding noise directly.

A large number of current research exploration methods that potentially set the exploration strategy *π*_*e*_ and action generation strategy *π* are highly similar and can be improved by applying various forms of random noise to the action generation strategy. However, this setting is not conducive to the expansion of state exploration. In contrast, the space that has not been explored in the past will be explored only when there is a significant difference between exploration strategy *π*_*e*_ and action generation strategy *π*. The amplitude of Gaussian noise is an important parameter that has been discussed for a long time, even in the method of using Gaussian noise as the exploration mode. Therefore, it is of great theoretical value and engineering significance to construct an adaptive exploration system method to replace the traditional probabilistic method.

As the DDPG algorithm is a typical off-policy learning method, its exploration process and learning process are independent from each other, so the exploration strategy *π*_*e*_ can be decoupled from the action generation strategy *π*. The specific idea is to construct a more efficient heuristic exploration strategy acting on the experience replay space to have a more positive role in the training of the action generation strategy *π*.

### 3.1. Algorithm Design

The framework proposed in this section can be regarded as a heuristic learning framework, in which the exploration strategy *π*_*e*_ acts as the heurist and generates a set of heuristic information *D*_0_ during each iteration, and the action generation strategy *π* learned by the DDPG algorithm acts as the heurist and receives the *D*_0_ heuristic strategy *π*_*e*_ and carries out training and learning. Therefore, the decisive factor is changed to adaptively improve the exploration strategy *π*_*e*_ to generate optimal value heuristic information *D*_0_ according to the learning efficiency of the DDPG algorithm so that DDPG can learn as quickly and effectively as possible.

The generation of heuristic information *D*_0_ can be considered as the action *a*_*e*_ performed by the exploration strategy *π*_*e*_, and its related reward function should be defined as the improvement of the DDPG algorithm through heuristic information *D*_0_:

(13) $$\begin{array}{c} J\left(\pi_{e}\right)=E_{D_{0}∼\pi_{e}}\left[R\left(\pi ,D_{0}\right)\right]\\ =E_{D_{0}∼\pi_{e}}\left[R_{\pi^{\prime }}-R_{\pi }\right], \end{array}$$

where *π*′=DDPG(*π*, *D*_0_) represents the new strategy obtained by one or more updated steps of the DDPG algorithm on the basis of heuristic information *D*_0_, *R*_*π*′_, and *R*_*π*_ represent the cumulative rewards of the DDPG algorithm obtained by strategy *π*′ and strategy *π* interaction with the environment, respectively, which have no relationship with exploration strategy *π*_*e*_. *R*(*π*, *D*_0_) represents the extent to which the heurist (exploration strategy *π*_*e*_) helps the heurist (DDPG algorithm) in the learning process.

Referring to the parameterized representation of the policy network in traditional DDPG, the policy *π*_*e*_ can be parameterized by parameters *θ*^*π*_*e*_^. Similar to the traditional reinforcement learning method, the gradient *J*(*π*_*e*_) of parameters *θ*^*π*_*e*_^ can be calculated as follows:

(14) $$\begin{array}{c} \nabla_{\theta^{\pi_{e}}}J\left(\pi_{e}\right)=E_{D_{0}∼\pi_{e}}\left[R\left(\pi ,D_{0}\right)\nabla_{\theta^{\pi_{e}}}\log\;P\left(D_{0}|\pi_{e}\right)\right], \end{array}$$

where *P*(*D*_0_*|π*_*e*_) represents the probability of generating heuristic information *D*_0_ : ={*s*_*t*_, *a*_*t*_, *r*_*t*_}_*t*=1_^*T*^ in the search strategy *π*_*e*_, and its distribution can be decomposed into

(15) $$\begin{array}{c} P\left(D_{0}|\pi_{e}\right)=p\left(s_{1}\right)\prod_{t=1}^{T}\pi_{e}\left(a_{t}|s_{t}\right)p\left(s_{t+1}|s_{t},a_{t}\right), \end{array}$$

where *p*(*s*_*t*+1_*|s*_*t*_, *a*_*t*_) is the state transition probability and *p*(*s*_1_) is the initial distribution. Since the probability *p*(*s*_*t*+1_*|s*_*t*_, *a*_*t*_) has no relationship with the exploration strategy parameters *θ*^*π*_*e*_^, a gradient of approximately *θ*^*π*_*e*_^ can be obtained as follows:

(16) $$\begin{array}{c} \nabla_{\theta^{\pi_{e}}}\log\;P\left(D_{0}|\pi_{e}\right)=\sum_{t=1}^{T}\nabla_{\theta^{\pi_{e}}}\log\;\pi_{e}\left(a_{t}|s_{t}\right). \end{array}$$

This value can be calculated from the data that the DDPG algorithm interacts with the environment.

To estimate the difference reward value *R*(*π*, *D*_0_), a heuristic strategy is adopted in this paper. The heuristic is realized by calling the DDPG algorithm one step or *n* steps in advance. First, a new action strategy is obtained by calling DDPG based on heuristic information *D*_0_, and then heuristic information is obtained by using the newly obtained action strategy *π*′=DDPG(*π*, *D*_0_). The cumulative reward value ${\hat{R}}_{\pi^{\prime }}$ of action strategy *π*′ can be estimated through heuristic information *D*_1_ so that the reward of travel value can be estimated as follows:

(17) $$\begin{array}{c} \hat{R}\left(\pi ,D_{0}\right)={\hat{R}}_{\pi^{\prime }}-{\hat{R}}_{\pi }, \end{array}$$

where ${\hat{R}}_{\pi }$ is the estimation of the reward function value of action strategy *π*, which is obtained by the previous iteration of the cycle.

After the difference reward *R*(*π*, *D*_0_) is obtained, the following parameters of the exploration strategy *π*_*e*_ are updated along the gradient direction of (16) by referring to the parameter *θ*^*π*_*e*_^ updating idea of the DDPG algorithm:

(18) $$\begin{array}{c} \theta^{\pi_{e}}\;⟵\;\theta^{\pi_{e}}+\eta \hat{R}\left(D_{0}\right)\sum_{t=1}^{T}\nabla_{\theta^{\pi_{e}}}\log\;\pi_{e}\left(a_{t}|s_{t}\right). \end{array}$$

After the exploration strategy *π*_*e*_ is updated, the heuristic information *D*_0_ and *D*_1_ are added to the experience replay space, that is, *B* ⟵ *B* ∪ *D*_0_ ∪ *D*_1_. The action strategy *π* is updated through the DDPG algorithm after sampling from the experience replay space, that is, *π* ⟵ DDPG(*π*, *B*). The specific Algorithm 1 process is as follows:

Although the improvement of the DDPG algorithm in this section increases the amount of computation in the calculation of heuristic data *D*_1_, the high efficiency *D*_1_ brought to the overall algorithm can compensate for this shortcoming. The construction of DDPG can not only be used to evaluate the improvement of learning performance but also participate in the update of action strategy *π*.

### 3.2. Performance Test of Algorithm

To test the performance of the improved algorithm proposed in this paper, Half Cheetah-v1, a Mujoco robot control environment in the OpenAI Gym toolkit, is selected as the test environment. Considering that the UCAV air combat in this paper is a decision-making process with air combat status information as input, without considering the image input, the RAM version of the environment is chosen and the state information is obtained directly, rather than the RGB version with the game graphics as input. To reflect the performance of the algorithm, 20 Monte Carlo simulations were performed for each algorithm. The *Q*(*s*_0_) curves of the three algorithms are shown in Figure 2.

In Figure 2, the ordinate ‘performance' is the cumulative reward value of completing a task. The areas covered by red, dark blue, and light blue are the heuristic DDPG algorithm proposed in this paper, the PPO algorithm and the traditional DDPG algorithm, respectively, after 20 Monte Carlo simulations of the *Q*(*s*_0_) distribution. The solid lines of the three colors are the average values of their distribution data. Through comparison, it can be seen that the heuristic DDPG algorithm has a stronger scoring ability after strengthening the exploration performance, which reflects a stronger ability to explore the optimal solution. Simulation comparison tests verify the effectiveness and superiority of the proposed algorithm.

## 4. Maneuver Decision Scheme Design

To increase the generalization ability of strategic networks, this paper considers the relative relationship between the enemy and the UCAV in the selection of state variables and takes the three-dimensional relative position coordinates of two aircraft, the relative flight speed, AA, and ATA as state variables; that is, the state variables are

(19) $$\begin{array}{c} s=\left[\Delta x,\Delta y,\Delta z,V,V_{e},\Delta V,\gamma ,\gamma_{e},\psi ,\psi_{e}\text{AA},\text{ATA}\right], \end{array}$$

where Δ*x*, Δ*y*, Δ*z* and Δ*V* are the relative position coordinates and relative flight speed of the two aircraft, respectively.

In the selection of the action, it is designed as the variation of the model control variable *u*=[*κ*, *α*, *ϕ*] of the UCAV platform in consideration of generating the smoothness of the maneuver trajectory.

(20) $$\begin{array}{c} a_{i}=\left[\Delta \kappa_{i},\Delta \alpha_{i},\Delta \phi_{i}\right], \end{array}$$

where Δ*κ*_*i*_, Δ*α*_*i*_, Δ*ϕ*_*i*_ represents the change in throttle lever, change in the angle of attack, and change in roll angle, respectively. The control variable *a*_*t*_ of the strategy network output at time *t* acts on the environment to produce the state *s*_*t*+1_ at the next step. Together with the state *s*_*t*_ at time *t*, the reward *r*_*t*_ constitutes the state transfer information [*s*_*t*_, *a*_*t*_, *r*_*t*_, *s*_*t*+1_].

## 5. Simulation and Analysis

### 5.1. Network and Parameter

Combined with the maneuver decision scheme, the actor network and critic network structures in our algorithm are designed. The structures of the actor network and actor target network are the same, and the input value is the state input *s*=[Δ*x*, Δ*y*, Δ*z*, *V*, *V*_*e*_, Δ*V*, *γ*, *γ*_*e*_, *ψ*, *ψ*_*e*_AA,ATA], so the input layer with 12 nodes is set. The output is the maneuvering action control variable *a*_*i*_=[Δ*κ*_*i*_, Δ*α*_*i*_, Δ*ϕ*_*i*_] in the current state; therefore, the number of nodes in the output layer is 3. The structure of actor network is shown in Table 1.

The critic network has the same structure as the critic target network. The input value is the combination of the state input *s*=[Δ*x*, Δ*y*, Δ*z*, *V*, *V*_*e*_, Δ*V*, *γ*, *γ*_*e*_, *ψ*, *ψ*_*e*_AA,ATA] and the change rate of the control value *a*_*i*_=[Δ*κ*_*i*_, Δ*α*_*i*_, Δ*ϕ*_*i*_] generated by the current actor network. Therefore, the input layer of 15 nodes is constructed, and the network output is the action value function Q. The structure of critic network is shown in Table 2.

The neural network training platform is a TensorFlow open-source deep learning computing platform based on an NVIDIA GeForce GTX 1080Ti GPU in an Ubuntu 16.04 system. The specific hyperparameter settings of the H-DDPG algorithm are shown in Table 3.

### 5.2. Initial Situation Setting

To verify the effectiveness of the algorithm, it is assumed that the enemy fighter and the UCAV adopt the same platform model and the same maneuverability constraints. The decision method of enemy adopts the rolling time-domain maneuver decision method proposed in reference [36]. In order to reflect the antagonism of air combat, we suppose the two sides enter the battle in a head-on encounter and set the UCAV height slightly lower than the enemy aircraft at a disadvantage. The simulation initialization state is shown in Table 4.

### 5.3. Enemy Making Random Maneuvers

**Case 1 .**

The UCAV weapon is stronger in the head-on situation, and the launching distance of the UCAV weapon is superior. The winning conditions of the UCAV are as follows: ATA ≤ 30°&200 m ≤ *D* ≤ 2500 m&0 m ≤ *h*_*r*_ − *h*_*b*_ ≤ 1000 m. The air battle trajectory is shown in Figure 3.

As shown in Figure 3, the enemy aircraft chooses to dive downward through a random maneuver. The UCAV approaches the enemy aircraft in flat flight and then dives downward to gain altitude superiority. It finally gives priority to meet the weapon firing conditions and launches missiles to win air battles. It can be seen from the changes of reward factors in Figure 4 that at the beginning of the battle, the UCAV had already met the maximum angle reward factor, approached the enemy aircraft through flat flight and dove at 21 s to obtain the height advantage, and reached the weapon launch range at 26 s. At this time, all the reward functions achieved 1, meeting the winning conditions in the air battle.  Figure 5 shows the curve of the average cumulative reward function value of training for this air combat mission. Each epoch on the horizontal axis contains 200 training missions, and the ordinate axis is the average cumulative reward value obtained for every 200 missions.

**Case 2 .**

The enemy weapon is stronger when the firing distance of the enemy weapon is dominant; the UCAV winning conditions are as follows: ATA ≤ 30°&AA ≥ 90°&200 m ≤ *D* ≤ 2500 m&0 m ≤ *h*_*r*_ − *h*_*b*_ ≤ 1000 m. Air battle trajectory is shown in Figure 6.

As seen from Figure 6, the enemy swooped down to the left through random maneuvers and then climbed to the left. Due to the low altitude at the beginning, the UCAV first shortened the distance with the enemy and improved the height advantage by climbing. Before entering the enemy attack range, it made a sharp right turn. The UCAV achieves a height advantage by successfully diving behind the enemy's tail and by turning to the right with a small overload. Finally, the UCAV achieves a height advantage by continuously following the enemy with a small overload deceleration and pulling up to the left to meet the rear attack conditions and win the air battle. As seen from the changes in reward factors in Figure 7, at the early stage of air combat, due to the long distance, low altitude, and enemy meeting the attack angle, all reward factors are −1. With the implementation of a large overload maneuver, the UCAV gradually obtains each situation advantage and finally meets the weapon launch conditions at 89 s by tracking the enemy aircraft. At the beginning of the battle, the UCAV has already met the maximum angle reward. It approaches the enemy through flat flight and dives at 21 s to gain an altitude advantage. At 26 s, the UCAV reaches the weapon launch range.  Figure 8 shows the curve of the cumulative reward value during the task training process in this section.

### 5.4. Enemy Making Intelligent Maneuvers

Under this task, the enemy makes intelligent maneuvers using the rolling time-domain maneuver decision method proposed in reference [36], which is adopted to traverse 216 trial maneuvers generated by the discrete variation of control variables, and the maneuvers corresponding to the optimal membership function value are selected and executed through the membership function of the air combat situation.

Mission setting: the enemy weapon is stronger. Under this mission, the UCAV adopts the rear attack mode to attack the enemy aircraft. The enemy does not need to go around the rear but adopts an omnidirectional attack strategy. The UCAV winning conditions are as follows: ATA ≤ 30°&AA ≥ 90°&200 m ≤ *D* ≤ 2500 m&0 m ≤ *h*_*r*_ − *h*_*b*_ ≤ 1000 m. After training, the maneuvering UCAV strategy gradually converges. Under this strategy, the air battle trajectory is shown in Figure 9.

As shown in Figure 9, after the two sides entered the air combat airspace in a head-on encounter, the enemy aircraft adopted an accelerated dive maneuver at a high altitude to quickly approach the UCAV to meet the priority conditions of weapon launch. The UCAV first adopted an accelerated flat flight to quickly shorten the distance between the two sides and pulled off to the upper left and right of the enemy aircraft before entering the enemy missile attack range. The enemy aircraft lost altitude advantage due to the rapid speed of the dive and then leveled out and pulled up to the left, regained altitude advantage and turned, but due to the climb maneuver reduced speed resulting in a larger turning radius. At this point, the UCAV performs a loop to increase its speed and power advantage and finally wins by following the enemy aircraft to reach the weapon firing conditions.

Figure 10 shows the reward function curve. It can be seen from the figure that in the 30 s–50 s range, the UCAV gained a temporary altitude advantage through a loop and then repositioned below the enemy aircraft until 105 s the UCAV remained level and dived, adjusting the angle by sacrificing its altitude advantage. After that, the UCAV succeeded in placing itself behind the enemy aircraft at 110 s gaining altitude and angle advantages. After that, the UCAV closed the distance by adjusting its attitude and defeated the enemy aircraft at 133 s.  Figure 11 shows the curve of control variable of UCAV.  Figure 12 shows the curve of the average cumulative reward value of training for this air combat mission. Each epoch on the horizontal axis contains 200 training missions, and the ordinate axis is the average cumulative reward value obtained for every 200 missions.

## 6. Conclusions

In this paper, a continuous action space air combat decision-making technology for UCAVs based on reinforcement learning is studied. Starting with the UCAV continuous action space model, a continuous action space air combat model is constructed based on the aerodynamic parameters of the unmanned stealth fighter. Focusing on the problems of weak exploration ability and low data utilization rate of the DDPG algorithm, a heuristic exploration strategy was introduced to propose a heuristic DDPG algorithm to improve the exploration ability of the original algorithm. The effectiveness and superiority of the proposed algorithm are verified by the Monte Carlo simulation in a typical continuous motion control environment (Half Cheetah). In the simulation verification stage, two subtasks with increasing difficulty, random maneuvers, and intelligent attack maneuvers are adopted for enemy aircraft, and the results show that the method presented in this paper can accomplish maneuver decisions under various tasks as well.

## Figures and Tables

**Figure 1:** Geometric relation of air combat position.

**Figure 2:** Comparison of the algorithm cumulative reward curve in the half Cheetah environment. (a) Half Cheetah environment interface. (b) Comparison of the algorithm cumulative reward curve.

**Figure 3:** Air combat trajectory. (a) 3D view of air combat trajectory. (b) Aerial view of the air combat trajectory. (c) Horizontal view of the air combat trajectory.

**Figure 4:** Curves of reward factors.

**Figure 5:** Cumulative reward curve.

**Figure 6:** Air combat trajectory. (a) 3D view of air combat trajectory. (b) Aerial view of the air combat trajectory. (c) Horizontal view of the air combat trajectory.

**Figure 7:** Curves of reward factors.

**Figure 8:** Cumulative reward curve.

**Figure 9:** Air combat trajectory. (a) 3D view of air combat trajectory. (b) Aerial view of the air combat trajectory. (c) Horizontal view of the air combat trajectory.

**Figure 10:** Curve of reward factors.

**Figure 11:** Curve of control variable. (a) Curves of the angle of attack and roll angle. (b) Curve of the throttle lever.

**Figure 12:** Curve of average cumulative reward.

**Algorithm 1:** Heuristic DDPG pseudocode.

**Table 1:** Actor/Actor target network structure.

Layer	Input	Activation function	Output
Input layer	1 × 12	None	128
Full connection layer 1	128	tanh	128
Full connection layer 2	128	tanh	128
Output layer	128	Linear	1 × 3

**Table 2:** Critic/Critic target network structure.

Layer	Input	Activation function	Output
Input layer	1 × 15	None	128
Full connection layer 1	128	tanh	128
Full connection layer 2	128	tanh	128
Output layer	128	Linear	1 × 1

**Table 3:** Hyperparameter setting of heuristic DDPG algorithm.

Parameter	Parameter value
Size of replay buffer *D*	50000
Size of minibatch *N*_*T*_	64
Actor learning rate *α*	0.0001
Critic learning rate *β*	0.001
Discount rate *γ*	0.99

**Table 4:** Initial state of UCAV and enemy.

	*x* (m)	*y* (m)	*z* (m)	*v* (m/s)	*γ* (°)	*ψ* (°)	Max step (s)
UCAV	0	0	10000	250	0	45	200
Enemy	10000	10000	12000	200	0	−135.	

## Data Availability

All data included in this study are available from the corresponding author upon request.
